RETRACTED

# Factors Analysis of the Compliance Rate of Hypertension Detection Control and Self-Assessment Control in Community Outpatient Clinics

**DOI:** 10.1155/2022/9432202

**Published:** 2022-10-12

**Authors:** Zhigao Chen, Rui Xiong

**Affiliations:** ^1^Hospital of Wuhan University of Science and Technology, Wuhan 430061, China; ^2^Wuchang District Shouyilu Street Community Health Service Center, Wuhan 430061, China

## Abstract

**Objective:**

To understand the related influencing factors of outpatient hypertension detection and control and self-test control compliance rate.

**Methods:**

A total of 637 hypertensive patients who visited the outpatient clinic of our hospital from January 2021 to December 2021 were selected for investigation and research, and the relevant information such as blood pressure, treatment detection, and other related information of the patients were counted, and the detection and control of outpatient hypertension were explored through regression analysis and the related factors of the self-test control compliance rate.

**Results:**

There was no statistically significant difference in the number of patients who met the standard or not under the gender difference (*P* > 0.05), and it can be found that there was no statistically significant difference in the age of patients who met the standard and those who did not (*P* > 0.05). The proportion of patients with self-test hypertension control at home was 64.68%, and the compliance rate of self-test blood pressure was 42.54%. The compliance rate of blood pressure control in outpatient testing was 61.85%. Heart rate, exercise, smoking, medication compliance, and other factors are important factors affecting the control of hypertension. Knowing hypertension-related knowledge, regular follow-up, office blood pressure compliance, smoking, excessive salt intake, and hypertension complications are important factors affecting the self-test control of hypertension in the family.

**Conclusion:**

By urging patients to do daily physical exercise, admonishing patients to quit smoking, and improving patients' medication compliance, the control rate of hypertension in outpatient clinics can be effectively improved. Understanding the knowledge of hypertension, controlling the salt content in the diet, and receiving regular follow-up surveys from doctors can effectively improve the effect of self-measurement and control of blood pressure at home and further improve the control rate of hypertension.

## 1. Introduction

At present, scholars have proved that bad habits such as smoking and drinking lead to poor blood pressure control in patients with hypertension. Family history of cardiovascular disease, long-term excessive drinking, smoking, diabetes, hyperlipidemia, and compliance with medical compliance are risk factors affecting blood pressure control in patients with hypertension. These factors should be paid attention to in clinical practice. But these studies are not in depth and need to be further explored.

RETRACTED

Hypertension is a common chronic disease, often accompanied by heart, kidney, and other target organ dysfunction or organic discoloration and is also a major risk factor for cardiovascular and cerebrovascular diseases such as stroke and coronary heart disease [1, 2]. In recent years, with the rapid improvement of the economic level, people's living patterns have changed, and the social population is aging. The fatality rate is also high, and it is one of the important causes of death [3–5]. Effective hypertension prevention and control is of great significance to reduce the prevalence and incidence of hypertension and can help hypertensive patients control their own blood pressure levels and improve their quality of life. In addition, the prevention and control of hypertension is also conducive to reducing the risk of related cardiovascular and cerebrovascular diseases and reducing people's disease burden.

Hypertension, as a common disease, seriously affected the physical condition of patients with hypertension. If the blood pressure of patients with hypertension is not well controlled, the increase in the range of blood pressure fluctuations can increase the cerebral perfusion pressure and lead to dizziness. Without timely treatment, it will even progress to small focal bleeding, causing amaurosis, or even fainting. Therefore, the common clinical symptoms of hypertension patients are dizziness, headache, blurred vision, blackening, and even fainting. Excessive drug dose in patients with hypertension may lead to low blood pressure. Similarly, insufficient cerebral perfusion can also cause transient ischemic attack, leading to dizziness, headache, and darkness. In severe cases, patients will also have symptoms of fainting. Low blood pressure caused by acute cerebral infarction will not only cause severe headaches but also cause coma [6].

Hypertension is a long-term chronic disease that requires patients to maintain long-term medication treatment to maintain a stable blood pressure state. Even if the patient's blood pressure level generally reaches the safe standard, there is still a certain residual risk of cardiovascular events [7, 8]. At present, the commonly used hypertension control method is a combined treatment mode including blood pressure monitoring, drug treatment, and life intervention, and strict blood pressure monitoring ensures stable blood pressure control of patients [9, 10]. Outpatient blood pressure testing can provide reference for doctors to diagnose and treat and provide accurate blood pressure data for patients. The economic cost and time cost of self-measurement of blood pressure at home are lower, and self-monitoring of blood pressure by patients outside medical institutions can effectively help hypertensive patients to quickly understand their blood pressure status in the home environment and prompt patients to take corresponding measures in a timely manner [11–13]. Therefore, the study analyzed the relevant factors of hypertension self-testing and the compliance rate of blood pressure detection and control in community outpatient clinics, in order to provide a reference for improving the blood pressure control compliance rate of hypertensive patients.

RETRACTED

Through the analysis of community outpatient hypertension detection control and self-test control compliance rate-related factors, we can more accurately grasp the blood pressure control of patients with hypertension to help patients with hypertension stable condition; normal life is of great significance.

## 2. Materials and Methods

### 2.1. General Information

The study cases were 637 hypertensive patients who visited the outpatient department of our hospital from January 2021 to December 2021. The inclusion criteria of the surveyed patients were as follows: (1) meet the diagnostic criteria of hypertension in the “Chinese Guidelines for the Prevention and Treatment of Hypertension 2010” and meet the systolic blood pressure ≥140 mmHg or diastolic blood pressure ≥90 mmHg. (2) Age >18 years old. (3) Have self-behavior, clear consciousness, and no communication barriers. The exclusion criteria are as follows: (1) patients with secondary hypertension. (2) Patients with severe cardiovascular and cerebrovascular complications in the past. (2) Suffering from mental illness and cognitive dysfunction. (3) Women who are pregnant or breastfeeding. All patients participated in the investigation and research voluntarily, and the patients and their families had signed the informed consent, and the research was approved by the ethics committee of our hospital. The general data of the study cases are shown in Table 1.

### 2.2. Research Methods

This study focuses on the analysis of the factors related to the compliance rate of hypertension detection control and self-test control in community clinics. On the premise of considering the age and gender factors of patients, the relevant evaluation criteria are measured by grouping patients in different groups. The effect of age on blood pressure control and the effect of gender on blood pressure control were also analyzed.

RETRACTED

The clinicians who have received unified training and passed the examination will conduct a questionnaire survey and physical examination on the subjects. They will learn about the age, disease, medication, physical exercise, family history, diabetes history, smoking and alcohol history, medication compliance, and other information of the subjects in the form of a questionnaire. After completing the questionnaire, they will review the questionnaire items in time and supplement the missing information. Physical examination included height, weight, and blood pressure measurements of the subjects. The height and weight of the subjects were measured according to standard methods. The subjects were required to take off their shoes and hats and wear single clothes. When measuring height, the subjects were required to stand barefoot close to the scale, keep their heels close together, and keep their shoulder blades, hips, and heels close to the scale. The height data reading was accurate to 0.1 cm. A platform scale was used to measure the weight of the subjects, and the weight data were accurate to 0.1 kg. The blood pressure of the subjects was measured according to the international common blood pressure measurement methods and quality control methods, and the standard mercury sphygmomanometer was used for measurement. Before the measurement, the subjects were required to sit and rest for at least 5 min and measure three times, ensuring that the interval between the two measurements was 1–2 min and taking the average value of the three measurements.

### 2.3. Judgment Criteria

In the examination of blood pressure in the consulting room, if the systolic blood pressure of the subjects under 60 years old is ≥ 140 mmHg or the diastolic blood pressure is ≥ 90 mmHg, the examination is unqualified. If the systolic blood pressure is ≥150 mmHg or diastolic blood pressure is ≥90 mmHg of subjects over 60 years old, the test is not up to the standard. In the family self-test, if the systolic blood pressure of the subject is ≥ 135 mmHg or the diastolic blood pressure is ≥ 85 mmHg, the test is unqualified. Salt intake ≥ 6G per day is considered as excessive salt intake. The study subjects who smoke or have quit smoking are smoking history, which refers to smoking and smoking more than 1 cigarette a day for more than 1 year or smoking more than 1 cigarette a day in the past but have quit smoking now. Drinking history refers to drinking more than 50 ml of baijiu, 150 ml of red wine, or 500 ml of beer every day. In the evaluation of physical exercise indicators, if the average number of exercises per week is ≥ 3 and the duration of each exercise is ≥ 30 min, it is judged that there is physical exercise. If the number of days of taking medicine according to the doctor's instructions exceeds 90% of the total number of days, it is judged that the medication compliance is good. Subjects with BMI ≥50 were obese, and BMI was the square of body weight divided by height.

RETRACTED

If the study object meets one of the conditions of plasma cholesterol rise ≥5.7 mmol/l, low-density lipoprotein cholesterol >3.6 mmol/l, or triglyceride rise ≥1.7 mmol/l, it is judged that the study object is dyslipidemia. The subjects with a history of typical angina pectoris and coronary artery stenosis ≥50% shown by coronary CTA or coronary angiography, or a history of myocardial infarction, were recorded as coronary heart disease. Cerebral hemorrhage and cerebral infarction were recorded as stroke complications, and heart failure included acute heart failure and chronic heart failure. If the daily urine protein quantity of the study object is more than 150 mg, or the urine protein qualitative test result is positive, or the urine protein/creatinine is more than 200 mg/g, the study object is judged to be proteinuria. Serum creatinine was higher than 133 umol/*L* in males and 124 umol/*L* in females. Left ventricular hypertrophy was diagnosed by the left ventricular mass index. If female ≥110 g/m^2^ and male ≥125 g/m^2^, left ventricular hypertrophy was judged. If there is atrial enlargement or left ventricular thickening in each atrium and ventricle of the study object, the study object is marked as cardiac enlargement and hypertrophy. If the carotid intima-media thickness of the subject is ≥ 1 cm, or there are single or multiple atherosclerotic plaques, the subject is marked as carotid artery thickening and plaque.

The above are diseases that interact with hypertension, but they are not comprehensive. If other diseases occur during the survey, they can be listed separately for analysis.

### 2.4. Statistical Analysis

Statistical software SPSS22.0 was used for data analysis, and measurement data were expressed as the mean ± standard deviation $\left(\bar{x}\pm s\right)$. Due to the large amount of data in the sample and all of them being numerical data, the average value of the sample variance can be calculated. Therefore, the *t*-test is used for intergroup comparison, the count data are compared between the groups by the test, and the related factors are analyzed by binary logistic stepwise regression. *P* > 0.05 indicates that the difference is statistically significant.

## 3. Results

### 3.1. Analysis of Related Factors of Hypertension Detection and Control

Table 2 shows the results of univariate analysis of blood pressure control in community outpatient clinics. Among 637 hypertensive patients, 394 had blood pressure control, and the compliance rate was 61.85%. The patients were grouped according to whether blood pressure detection and control reached the standard. It can be seen that the difference in the number of people who reached the standard or not under the gender difference was not statistically significant (*P* > 0.05). There were statistically significant differences between those who reached the standard and those who did not reach the standard under such indicators as BMI, heart rate, exercise, smoking, drinking, medication compliance, and excessive salt intake (*P* < 0.05).

RETRACTED

The multivariate analysis results of the influencing factors of hypertension detection and control are shown in Table 3. Logistic regression analysis was used to evaluate the degree of influence of the indicators. Whether the patient's control was up to the standard was used as the dependent variable, and BMI, heart rate, exercise, smoking, drinking, and medication were used as the dependent variable. The factors affecting compliance and excessive salt intake, namely independent variables, were analyzed by logistic regression. The results showed that the multivariate analysis *P* value of the heart rate, exercise, smoking, and medication compliance was less than 0.05, indicating that factors such as the heart rate, exercise, smoking, and medication compliance were important influencing factors for hypertensive patients to be controlled. It is a risk factor for hypertension control, and regular exercise and high medication compliance are protective factors for hypertension control.

The ROC curve is used to reflect the diagnostic performance of the heart rate, exercise, smoking, and medication compliance indicators in hypertension clinics. The OR value of the heart rate was 0.997, between 0.824 and 1.039, so heart rate block was a risk factor for high snow pressure control. Smoking is also a risk factor for blood pressure control. Conversely, exercise and medication adherence are protective factors for blood pressure control. The ROC curve of the heart rate, exercise, smoking, and medication compliance in the prediction of blood pressure control compliance in patients with hypertension is shown in Figure 1, and the areas under the ROC curve of the heart rate, exercise, smoking, and medication compliance were 0.779, 0.752, 0.821, and 0.704, respectively.

### 3.2. Analysis of Influencing Factors of Self-Assessment and Control of Hypertension

The results of blood pressure self-testing in community outpatient clinics are shown in Table 4. Among 637 hypertensive patients, 412 had self-measured blood pressure, and 225 had not performed home blood pressure self-measurement. Grouped by educational background, 51.71% of hypertensive patients with primary school and below took blood pressure self-testing at home, and 71.88% of hypertensive patients with high school education or above took home self-testing; the proportions of hypertensive patients with failure and dyslipidemia were 38.26%, 39.81%, and 32.93%, respectively; the proportion of hypertensive patients with a history of hypertension at home was 91.54%. 49.77% of hypertensive patients with no history of hypertension had self-measured blood pressure at home.

RETRACTED

Table 5 shows the results of univariate analysis of blood pressure self-assessment and control compliance, in which the number of blood pressure self-assessment compliance was 271, and the compliance rate was 42.54%. Gender, age, and occupation had no significant effect on the number of hypertensive patients who met the control standard at home (*P* > 0.05); hypertension, smoking, drinking, salt intake, follow-up, sleep quality, exercise, and hypertension complications were investigated; there was a statistically significant difference between the number of people who reached the standard and those who did not meet the standard of target organ damage and outpatient blood pressure (*P* < 0.05). Thus, education has a significant impact on home control of hypertension (*P* < 0.05), complications of hypertension also have a significant impact on home control of hypertension (*P* < 0.05), and the same history of hypertension in parents also has a significant impact on home control of hypertension. (*P* < 0.05).

Logistic regression analysis was used to determine the main influencing factors that affect the self-assessment and control of hypertension. The multivariate analysis results of the self-assessment and control of hypertension are shown in Table 6. Knowledge of hypertension, regular follow-up, and meeting the blood pressure in the office are the most important factors for family high blood pressure. The protective factors of blood pressure self-assessment and control, smoking, high salt intake, and hypertension complications are the risk factors for family blood pressure self-assessment and control.

The ROC curve is used to reflect the knowledge about hypertension, regular follow-up, meeting the blood pressure in the office, exercise, smoking, high salt intake, and suffering from hypertension complications. The ROC curve of the main factors controlling the compliance is shown in Figure 2. The areas under the ROC curve of knowledge of hypertension, regular follow-up, standard office blood pressure, smoking, excessive salt intake, and hypertension complications were 0.719, 0.704, 0807, 0.725, 0.694, and 0.757.

RETRACTED

## 4. Discussion

Hypertension is a common disease among middle-aged and elderly people. The occurrence of hypertension can lead to cardiovascular diseases such as myocardial failure and cerebral apoplexy in the middle-aged and elderly, which seriously endangers the normal life of middle-aged and elderly people [14, 15]. For hypertensive diseases, drug therapy is a common basic treatment method for hypertensive patients, but the role of drug therapy alone in blood pressure control is limited. For this reason, in order to improve the effect of hypertension control, it is important to understand the relevant factors affecting hypertension control [16, 17]. In medical research, it is found that the detection and control of hypertension includes two ways: outpatient hypertension detection and control and patient self-test control at home. In general, outpatient hypertension detection and control is to use drugs to help patients suppress blood pressure, and self-test control of blood pressure at home is to promote patients to change bad habits in daily life by improving patients' cognition of hypertension. Drug therapy and living habits play a supporting role in taking medicine while developing a good life schedule, such as getting up early and going to bed and exercising actively, can help patients with hypertension in better recovery. In general, outpatient hypertension detection and control is to use drugs to help patients suppress elevated blood pressure. Home blood pressure self-test control is to promote patients to change bad habits in daily life by improving their awareness of hypertension [18, 19]. Medication and lifestyle habits play an auxiliary role in taking medication, while making a good life plan, such as getting up early and going to bed, and taking active exercise, can help people with hypertension recover better. In general, outpatient hypertension detection and control is to use drugs to help patients suppress blood pressure rise, and home blood pressure is automatically controlled. Measurement and control is to promote patients to change their bad habits in daily life by improving their awareness of hypertension [18, 19]. Therefore, in order to effectively control blood pressure in hypertensive patients, the study starts from two aspects of outpatient detection and control and home self-measurement control, and it analyzes the relevant factors that affect outpatient detection and control and self-measurement control treatment and control rates [20].

The study conducted an analysis of the compliance rate of hypertension outpatient testing and control in community outpatient clinics. The results showed that the blood pressure control compliance rate in outpatient testing was 61.85%. Through univariate analysis, it was concluded that BMI, heart rate, exercise, smoking, drinking, medication compliance, and excessive salt intake can affect the compliance rate of outpatient hypertension detection and control. Multivariate logistic regression analysis showed that the rapid heart rate and smoking were risk factors for hypertension control, while regular exercise and high medication compliance were protective factors for hypertension control. The increased heart rate can lead to an excited state of the sympathetic nerves, which promotes the production of thyroxine, which in turn causes the arterioles to constrict and raise blood pressure [21–23]. Smoking stimulates the central and sympathetic nerves, which in turn promotes the contraction of small arteries and increases blood pressure. Exercise is an important way to improve personal physical fitness. Exercise can relax the patient's mood, reduce abnormal vasoconstriction caused by emotional stress, and reduce the probability of blood pressure increase [24, 25]. Medication compliance can help patients use antihypertensive drugs regularly, reduce the occurrence of drug side effects, and achieve the effect of blood pressure control, which is consistent with previous research results [26–28]. At the same time, there is also an interaction effect between them. Active exercise and taking drugs will have a positive feedback effect. There is a negative feedback effect between taking drugs and smoking and the increased heart rate. In other words, smoking and the increased heart rate will reduce the effect of drugs, while active exercise will make the effect of drugs better. Therefore, in the detection and control of hypertension in outpatient clinics, instructing patients to quit smoking, exercising more, and taking medicine regularly can improve the effect of blood pressure control and improve the quality of life of patients [29].

RETRACTED

The study showed that 64.68% of the experimental subjects took home self-measured hypertension control, and the self-measured blood pressure compliance rate was 42.54%. Through univariate analysis, the influencing factors of hypertension patients' self-measured blood pressure at home included hypertension-related knowledge, smoking, drinking, salt intake, follow-up, sleep quality, exercise, hypertension complications, and outpatient blood pressure compliance. Multivariate analysis was performed to determine the risk factors affecting the self-measured blood pressure control of patients. Using multivariate logistic regression analysis, the results showed that smoking, excessive salt intake, and suffering from hypertension complications were the risk factors for home hypertension self-assessment control. Knowledge of hypertension, regular follow-up, and meeting the standard of blood pressure in the office are the protective factors for the self-measured control of hypertension at home. It is known from numerous studies that increased salt intake can lead to increased water and sodium retention in the body, which in turn can lead to increased blood pressure. Hypertensive complications are malignant consequences of hypertension, and hypertensive complications can also feedback the status of hypertension, further aggravating the condition of hypertension [30–32]. For patients with hypertension at home, their awareness of hypertension is the basis for prompting patients to reasonably control their hypertension. Regular follow-up by doctors can help patients conduct regular monitoring and control. In addition, meeting the standard of blood pressure detection in the office can help patients with hypertension to scientifically control their hypertension. Knowing the status of their own blood pressure control will also induce patients to measure their blood pressure control at home [33, 34]. The above results show that for hypertensive patients who control their blood pressure at home, they need to reduce the frequency of smoking, control their diet, and pay attention to their own hypertension complications. They also need to participate in surveys of regular follow-up visits by physicians.

To sum up, in the detection and control of hypertension, urging patients to participate in daily physical exercise, admonishing patients to quit smoking, and improving medication compliance can improve the control rate of hypertension in outpatient clinics. Blood pressure and regular follow-up surveys by doctors can effectively improve the control effect of blood pressure self-measurement at home in hypertensive patients and further improve the control rate of hypertension. There are still some limitations in the study. The selection of hypertensive patients is affected by regional and cultural factors, which makes the selection of relevant factors difficult to be universal. Therefore, in the follow-up research, the research scope needs to be gradually expanded, and the detection and control of hypertension should be discussed in depth.

This study starts with a large amount of data and studies the factors related to the compliance rate of hypertension detection control and self-test control in community clinics under the premise of eliminating gender factors, age factors, complication factors, family history factors, and others. It has great research significance and has a significant effect on improving the self-behavior management and quality of life of patients with hypertension. There are still some limitations in the study. There are regional cultural factors in the selection of hypertension patients, which makes the selection of relevant factors difficult to have universality. Therefore, in the follow-up study, the scope of the study needs to be gradually expanded, and the risk factors and protective factors of hypertension detection and control are discussed in depth.

RETRACTED

## Figures and Tables

**Figure 1:** ROC curve of risk factors for hypertension detection.

**Figure 2:** Multifactor ROC curve of hypertension self-assessment and control compliance.

**Table 1:** General information (*n* = 637).

Variable		Number of cases	Composition ratio (%)
Gender	Male	267	41.92
	Female	365	58.08
Age	60≤, <70	308	48.35
	≥70	329	51.65
Educational level	Elementary school and below	381	59.81
	Secondary school and above	256	40.19
BMI	Normal	174	27.32
	Overweight	463	72.68
Family history	Parents with high blood pressure	201	31.55
	Parents without hypertension	436	68.45
Smoking history	Yes	367	57.61
	No	270	42.39
Hypertension comorbidities	Stroke	264	41.44
	Heart failure	206	32.34
	Dyslipidemia	167	26.53
Target organ damage	Cardiac enlargement and hypertrophy	213	33.44
	Carotid artery thickening and plaque	197	30.93
	Proteinuria and elevated serum creatinine	227	35.64

**Table 2:** Univariate analysis results of outpatient hypertension detection and control.

Variable		Up to standard ($\bar{x}\pm s$, *n*)	Not to standard ($\bar{x}\pm s$, *n*)	t/*χ*^2^	*P*
Gender	Male	196 (49.75%)	119 (48.97%)	0.139	0.772
	Female	198 (50.25%)	124 (51.03%)		
Age		66.37 ± 10.62	66.83 ± 10.24	0.543	0.587
BMI (kg/m^2^)		24.65 ± 3.31	24.53 ± 3.33	2.395	0.017
Heart rate (times/min)		75.31 ± 5.54	76.36 ± 5.71	2.280	0.023
Exercise	YES	189 (47.97%)	97 (39.92%)	8.269	0.004
	NO	205 (52.03%)	146 (60.08%)		
Smoking	YES	216 (54.82%)	155 (63.79%)	21.064	0.001
	NO	178 (45.18%)	88 (36.21%)		
Drinking	YES	117 (29.70%)	132 (54.32%)	10.617	0.001
	NO	277 (70.30%)	111 (45.68%)		
Medication compliance	GOOD	381 (96.70%)	192 (79.01%)	28.643	0.001
	LACK	13(3.30%)	51(20.99%)		
Excessive salt intake	YES	372 (94.42%)	232 (95.47%)	5.024	0.025
	NO	22 (5.58%)	11 (4.53%)		

**Table 3:** Multivariate logistic analysis results of outpatient hypertension detection and control.

Elements	*β*	*SE*	Wald *χ*^2^	*P*	*OR* (95%*CI*)
Heart rate	0.059	0.031	10.352	0.002	0.997 (0.824–1.039)
Exercise	0.972	0.442	15.776	0.001	0.325 (0.303–0.464)
Smoking	0.936	0.439	32.364	0.001	2.579 (1.929–3.816)
Medication compliance	1.157	0.507	44.853	0.001	0.153 (0.127–0.221)

RETRACTED

**Table 4:** Data of patients with hypertension controlled by self-testing at home.

project	Education		Hypertension complications			Parental history of hypertension	
	Elementary school and below	Secondary school and above	Stroke	Myocardial failure	Dyslipidemia	Yes	No
Self-test	197 (51.71%)	184 (71.88%)	101 (38.26%)	82 (39.81%)	55 (32.93%)	184 (91.54%)	217 (49.77%)
Not self-tested	184 (48.29%)	72 (28.12%)	163 (61.74%)	124 (60.19%)	112 (67.07%)	17 (5.46%)	219 (50.23%)
*χ* ^2^	10.127		8.523			14.339	
*P*	<0.05		<0.05			<0.05	

**Table 5:** Univariate analysis results of hypertension self-assessment and control compliance

Variable		Up to standard($\bar{x}\pm s$, *n*)	Not to standard($\bar{x}\pm s$, *n*)	t/*χ*^2^	*P*
Gender	Male	138 (49.08%)	72 (51.06%)	0.139	0.772
	Female	133 (50.902%)	69 (48.94%)		
Age		66.26 ± 10.72	66.65 ± 10.57	0.543	0.587
Profession	Brain power	127 (46.86%)	63 (44.68%)	1.264	0.642
	Physical strength	144 (53.14%)	78 (55.32%)		
Exercise	Yes	103 (38.01%)	52 (36.88%)	8.269	0.004
	No	168 (61.99%)	89 (63.12%)		
Smoking	Yes	113 (41.70%)	61(43.26%)	21.064	0.001
	No	158 (58.30%)	80 (56.74%)		
Drinking	Yes	117 (43.17%)	63 (44.68%)	10.617	0.001
	No	154 (56.83%)	78 (55.32%)		
High blood pressure-related knowledge	Know	126 (46.49%)	43 (30.50%)	28.643	0.001
	Do not know	145 (53.51%)	98 (69.50%)		
Excessive salt intake	Yes	142 (52.40%)	88 (62.41%)	5.024	0.025
	No	129 (47.60%)	53 (37.59%)		
Follow-up	Regular	163 (60.15%)	79 (56.03%)	10.332	0.037
	Irregular	108 (39.85%)	62 (43.97%)		
Sleep quality	Good	123 (45.39%)	59 (15.60%)	6.727	0.029
	Poor	148 (54.61%)	82 (58.16%)		
Hypertension complications	Yes	192 (70.85%)	141 (84.40%)	12.369	0.007
	No	79 (29.15%)	22 (15.60%)		
Target organ damage	Heart enlargement and hypertrophy	81 (29.15%)	51 (29.89%)	9.379	0.014
	Carotid thickening and plaque	93 (34.32%)	42 (15.80%)		
	Proteinuria, increased serum creatinine	97(35.79%)	48(17.71%)		
Office blood pressure up to the standard	Yes	194 (71.59%)	78 (55.32%)	5.337	0.009
	No	77 (28.41%)	63 (44.68%)		

**Table 6:** Multivariate analysis results of self-assessment and control in hypertensive patients.

elements	*β*	*SE*	Wald *χ*^2^	*P*	*OR* (95%*CI*)
Smoking	0.574	0.298	8.185	0.002	0.543 (0.264–0.710)
Office blood pressure up to the standard	1.072	0.556	12.349	0.001	1.201 (0.915–1.318)
Know about high blood pressure	0.825	0.407	5.446	0.005	0.526 (0.415–0.618)
Excessive salt intake	0.092	0.047	15.299	0.007	0.235 (0.129–0.307)
Regular follow-up	1.123	0.784	7.553	0.001	0.997 (0.829–1.054)
Have high blood pressure	1.256	0.539	11.265	0.005	1.127 (1.063–1.198)

## Data Availability

The datasets used and/or analyzed during the current study are available from the corresponding author on reasonable request.
